# The intratumoral microbiota: a new horizon in cancer immunology

**DOI:** 10.3389/fcimb.2024.1409464

**Published:** 2024-07-29

**Authors:** Wei Liu, Yuming Li, Ping Wu, Xinyue Guo, Yifei Xu, Lianhai Jin, Donghai Zhao

**Affiliations:** ^1^ College of Laboratory Medicine, Jilin Medical University, Jilin, China; ^2^ General Surgery Department of Liaoyuan Central Hospital, Jilin, China; ^3^ Low Pressure and Low Oxygen Environment and Health Intervention Innovation Center, Jilin Medical University, Jilin, China; ^4^ College of Basic Medicine, Jilin Medical University, Jilin, China

**Keywords:** intratumoral microbiota, immunotherapy, tumor immune microenvironment, immunomodulation, heterogeneity

## Abstract

Over the past decade, advancements in high-throughput sequencing technologies have led to a qualitative leap in our understanding of the role of the microbiota in human diseases, particularly in oncology. Despite the low biomass of the intratumoral microbiota, it remains a crucial component of the tumor immune microenvironment, displaying significant heterogeneity across different tumor tissues and individual patients. Although immunotherapy has emerged a major strategy for treating tumors, patient responses to these treatments vary widely. Increasing evidence suggests that interactions between the intratumoral microbiota and the immune system can modulate host tumor immune responses, thereby influencing the effectiveness of immunotherapy. Therefore, it is critical to gain a deep understanding of how the intratumoral microbiota shapes and regulates the tumor immune microenvironment. Here, we summarize the latest advancements on the role of the intratumoral microbiota in cancer immunity, exploring the potential mechanisms through which immune functions are influenced by intratumoral microbiota within and outside the gut barrier. We also discuss the impact of the intratumoral microbiota on the response to cancer immunotherapy and its clinical applications, highlighting future research directions and challenges in this field. We anticipate that the valuable insights into the interactions between cancer immunity and the intratumoral microbiota provided in this review will foster the development of microbiota-based tumor therapies.

## 1 Introduction

For a long period, it was widely believed that the tumor interior was a sterile environment. It wasn’t until the early 21st century, with the advancement of high-throughput sequencing technologies, that we were able to thoroughly investigate the microbiota within tumor tissues (Knippel et al., 2021; Sholl et al., 2022). In a global study, Nejman et al. conducted 16S rRNA sequencing on 1,010 tumor specimens and 516 adjacent non-tumor specimens from seven cancer types. They discovered that all of these cancer types, including ovarian cancer, glioma, and osteosarcoma, harbored DNA from bacteria that are not directly exposed to the external environment, and that each type of tumor exhibited a unique microbiota composition. This study opened a new chapter in the field of intratumoral microbiota research (Nejman et al., 2020).

Subsequent extensive research has confirmed the presence of microbiota in various types of cancer. Microbiota within tumors have long been recognized as a significant component of the tumor microenvironment (TME) (Dudgeon and Dunkley, 1907; Epstein et al., 1964; Warren and Marshall, 1983; Wotherspoon et al., 1991). Researchers now recognize the critical role of the intratumoral microbiota-driven host-tumor immune responses in influencing the efficacy of cancer immunotherapy (Matson et al., 2021). However, the impacts of microbiota that have colonized different tissues and organs on TME vary significantly. The gut barrier provides the largest host-microbiota interface and the greatest microbial diversity. Currently, research on the causal relationship between intratumoral microbiota and tumor immune responses primarily focuses on the gut microbiota. Derosa et al. systematically elucidated the relationships between distinct gut bacteria and local or systemic immune responses, summarizing tumor treatment interventions based on the gut microbiota (Derosa et al., 2021). Pham et al. summarized the relationships between the composition of the gut microbiota or microbiota-derived metabolites and the response to immune checkpoint blockade (ICB) therapy, proposing various strategies to modulate the microbiota composition within patients to enhance ICB efficacy and reduce adverse effects (Pham et al., 2021). The gut microbiota can utilize its components or metabolites to modulate tumor immunity, extending from the initial location in the gut to distant organs (Aghamajidi and Maleki Vareki, 2022; Lu et al., 2022; Ozcam and Lynch, 2024). However, it is noteworthy that extragastrointestinal tumors each possess their own microbiota, with distinct impacts on systemic immunity and the immune microenvironment that influence the progression of various types of tumors (Liang et al., 2023). It is essential to comprehensively explore the complex interactions among microbiota and host immune responses to elucidate the effects of tumor immunotherapy. Existing studies lack a systematic summary of the relationships among extragastrointestinal tumor microbiota and immune responses. Therefore, this review summarizes the intricate relationships between tumor immunity and intratumoral microbiota, both within and outside the gut, and attempts to explore their potential associations with tumor immunotherapy. Finally, based on our extensive research in these areas, we aim to promote the development of personalized strategies for tumor immunotherapy, ultimately improving treatment outcomes for cancer patients.

## 2 Genesis of intratumoral microbiota

The microbiota present within tumor tissues comprising the TME are collectively referred to as the intratumoral microbiota, and include bacteria, fungi, viruses, and mycoplasmas (Tang et al., 2013; Aykut et al., 2019; Poore et al., 2020). So far, microbiota have been detected in over 20 types of malignant tumors. There are four potential routes through which microbiota reach the intratumoral space: (1) resident microbiota originating in the same tissue where the tumor arises; (2) bloodstream transport of microbiota to the tumor site, a process that may also accompany cancer cell metastasis; (3) retrograde flow of gut microbiota through the common bile duct, common hepatic duct, and main pancreatic duct to tumor sites in the liver, bile ducts, and pancreas; and (4) oral-derived microbiota (**Figure 1**).

**Figure 1:** Elucidating the genesis of intratumoral microbiota, including: resident microbiota originating in tumors, the microbiota conveyed by the blood circulatory system, oral-derived microbiota and retrograde flow of gut microbiota. Graphics created with figdraw.com.

## 3 Heterogeneity of the intratumoral microbiota

There is considerable heterogeneity in the composition and abundance of the intratumoral microbiota across different tumor types. This heterogeneity arises from the distinct native microbiota of each organ, symbiotic microbiota entering the tumor site through various routes, and interactions between the TME and intratumoral microbiota. Current studies indicate that microbial distribution varies significantly among different tumor types, and the intratumoral microbial landscape may also differ among various subtypes of the same tumor. The composition of the intratumoral microbiota is predominantly bacterial, with lower relative abundances of fungi and mycoplasmas (Narunsky-Haziza et al., 2022). Xue et al. used 16S rRNA gene sequencing to reveal that the most abundant microbial genera in pancreatic cancer patients were found among *Proteobacteria*, *Bacteroides*, and *Firmicutes*. In colorectal cancer (CRC) tissues, there was enrichment of *Fusobacterium* and *Bifidobacterium*. Inflammatory bacteria, such as *Fusobacterium nucleatum* and *Pseudomonas aeruginosa*, were significantly predominant in oral squamous cell carcinoma (OSCC) tissues. Ovarian cancers exhibited a high proportion of human papilloma virus (HPV)-positive cells, while breast cancer tissues contained relatively low levels of bacteria (Xue et al., 2023). Guo et al. analyzed the intratumoral microbiota of 62 patients with pancreatic ductal adenocarcinoma (PDAC) and found that *Acinetobacter*, *Pseudomonas*, and *Sphingomonas* were highly associated with tumorigenesis and had the potential to induce inflammation, leading to carcinogenesis (Guo et al., 2021). Minarovits et al. discovered that, compared to normal colon tissues, CRC tissues harbored higher abundances of microbiota including *F. nucleatum*, *Fusobacterium periodonticum*, *Gemella morbillorum*, and *Peptostreptococcus stomatis* (Minarovits, 2021). Conde-Perez et al. analyzed the microbiota of saliva, gingival crevicular fluid, feces, and non-tumor and tumor intestinal tissue samples from 93 CRC patients and 30 healthy individuals without digestive system diseases. They developed an excellent noninvasive fecal detection method for early diagnosis of CRC using a label design composed of the genera *Bacteroides*, *Acinetobacter*, *Pseudomonas*, and *Clostridium* (Conde-Perez et al., 2024). A microbiomic study of mouthwash samples from 51 healthy individuals and 197 OSCC patients at different stages reconfirmed the association of the phylum Fusobacteria with this type of carcinoma (Yang et al., 2018). Nicolaro et al. found a close association between *Schistosoma haematobium* infection and the high incidence of bladder cancer (Nicolaro et al., 2020). In epithelial cells of lung cancers, microbiota including *P. aeruginosa, Streptococcus pneumoniae*, and other *Streptococcus* spp. were found to modulate the ERK and PI3K signaling pathways, which have been implicated in the development of non-small cell lung cancer (NSCLC) (Tsay et al., 2018).

## 4 Carcinogenesis of the intratumoral microbiota

Several primary modes of interaction may exist between the intratumoral microbiota and developing cancer (Garrett, 2015): (1) promotion of tumorigenesis via increases in host genomic instability and mutations, such as the DNA damage induced by the colibactin toxin of polyketide synthase (pks)+ strains of *Escherichia coli*, which lead to CRC (Chen et al., 2023); (2) regulation of tumor cell signal transduction, in which microbiota such as *Helicobacter pylori* and *F. nucleatum* are thought to mediate the Wnt/β-catenin pathway to promote cancer formation (Buti et al., 2011; Rubinstein et al., 2013; Wang et al., 2023); (3) tumor progression influenced by modulation of the host immune system, with studies indicating that intratumoral microbiota induce pro-inflammatory responses and promote tumor proliferation through activation of the NF-κB or STAT3 pathways (Bhatt et al., 2017, Garrett, 2015); (4) regulation of tumorigenesis, metastasis, and drug resistance through metabolic products, as evidenced by the Fu et al. study showing that intratumoral bacteria can enhance the resistance of host cells to mechanical stress from blood flow, thereby promoting breast cancer metastasis (Fu et al., 2022); and (5) modulation of the epigenetic status of tumor cells, particularly in gastric cancer, where intratumoral microbiota such as *Kytococcus sedentarius* and *Actinomyces oris* are significantly associated with methylation changes in immune-related genes of cancer cells, thus affecting gene expression (Yue et al., 2023).

## 5 Effects of the intratumoral microbiota on the tumor immune microenvironment

The TIME has been likened to a battlefield of tumor immune promotion and inhibition, playing crucial roles in tumor initiation, development, metastasis, and response to treatment. One of the most notable features of the intratumoral microbiota is its vulnerability to surveillance and recognition by the immune system, thereby triggering specific immune responses (Cogdill et al., 2018). The intratumoral microbiota shapes and regulates the TIME via several mechanisms: In the first mechanism, activation of inflammatory signaling pathways and release of cytokines via interactions with pattern recognition receptors (PRRs), such as Toll-like receptors (TLRs), affects the recruitment, maturation, and function of immune cells (Abreu and Peek, 2014; Hoste et al., 2015; Rutkowski et al., 2015; Pushalkar et al., 2018; Liwinski et al., 2020; Zhang et al., 2021). For example, *F. nucleatum* promotes the expression of CCL20 in tumor cells in CRC, inducing the polarization of M2 macrophages and enhancing the metastatic ability of cancer cells (Xu et al., 2021). The second mechanism involves regulation of tumor immunity through metabolites, with Luu et al. demonstrating that short-chain fatty acids such as valerate and butyrate enhance the antitumor activities of CTLs and CAR-T cells through metabolic and epigenetic reprogramming (Luu et al., 2021). Promotion of tumor-associated inflammation, in which chronic inflammation caused by long-term microbial infection in the TME contributes to tumor development and immune evasion, is the third mechanism. *F. nucleatum*, for example, is considered an immune-suppressive microbe that can induce the release of large amounts of inflammatory factors (Gur et al., 2015). The fourth mechanism involves microbes altering the physical properties of the TME, such as the pH or oxygen concentration, through the production of exogenous substances. These physical changes can impact the function of immune cells and the behavior of tumor cells.

The intratumoral microbiota also regulates host tumor immunity through various mechanisms. Some microbiota activate the host immune system to enhance immune surveillance of the tumor, while others help tumor cells escape immune system attacks by inducing immune tolerance or activating immunosuppressive pathways.

Mechanisms by which intratumoral microbiota enhance antitumor immune responses include the following. The first mechanism involves regulation of tumor immune responses through various signaling pathways, including the ROS, β-catenin, TLR, ERK, NF-κB, and STING pathways. Lam et al. demonstrated that the intratumoral microbiota modulates the pro-tumor/anti-tumor balance within the TIME through a STING-IFN I-dependent mechanism, reprogramming intratumoral macrophages to promote antitumor immunity and the efficacy of ICB therapy (Lam et al., 2021). In another example, enterogenic *Bacteroides fragilis* toxin degrades E-cadherin and activates β-catenin, promoting CRC formation by amplifying Tregs and Th17 cells (Sears and Garrett, 2014). The activation of T cells and NK cells mechanism includes bacteria in melanoma that activate DCs, thereby triggering T cells immune responses (Choi et al., 2023). In other examples, metabolites of *Lactobacillus plantarum* L168, such as I3A, improve colorectal tumorigenesis through epigenetic regulation of CD8+ T-cell immunity (Zhang et al., 2023), while clinical outcomes in patients with HPV-positive OSCC are superior to those with HPV-negative cancer, attributable to the presence of higher numbers of infiltrating IFNγ+CD8+ T lymphocytes, IL-17+ CD8+ T lymphocytes, myeloid DCs, and pro-inflammatory chemokines (Partlova et al., 2015). The third and fourth mechanisms involve formation of tertiary lymphoid structure (TLS) and enhancement of antigen presentation, respectively. In the latter, peptides from intratumoral bacteria are presented by antigen-presenting cells to further activate tumor-specific T-cell responses. An analysis of 17 melanoma metastases revealed 283 unique human leukocyte antigen (HLA)-I and HLA-II peptides derived from 41 different bacterial species. Recurrent bacterial peptides were identified in tumors from different patients as well as in different tumors from the same patient (Kalaora et al., 2021). Secretion of vesicles is the fifth mechanism, as shown by Kim et al., who discovered that outer membrane vesicles (OMVs) obtained from Gram-negative bacteria possess the ability to induce the production of cytokines CXCL10 and IFN-γ, thereby generating long-term antitumor immune responses (Kim et al., 2017) (**Figure 2**).

**Figure 2:** The intratumoral microbiota orchestrates a complex modulation of immune regulatory mechanisms within the tumor. Graphics created with figdraw.com.

Mechanisms by which intratumoral microbiota promote tumor development through inflammation or immune dysregulation include the following. The first is upregulation of ROS, as exhibited by *F. nucleatum*, which induces impairment of autophagic flux, enhancing the expression of proinflammatory cytokines via ROS in adenocarcinoma cells (Tang et al., 2016). The second mechanism involves modulation of cytokine production. Tipα of *H. pylori* stimulates the secretion of TNF-α and chemokines via the NF-κB signaling pathway, promoting gastric cancer development (Suganuma et al., 2012). Utilizing *in situ* spatial profiling and single-cell RNA sequencing techniques, invasive bacteria were shown to recruit bone marrow cells in oral squamous cell carcinoma and CRC, inducing inflammation through the JAK-STAT signaling pathway and promoting tumor growth by secreting interleukins and chemokines (Galeano Nino et al., 2022). Inhibition of T cells and NK cells activity is the third mechanism, as evidenced by direct interaction between the Fap2 protein of *F. nucleatum* and the inhibitory receptor TIGIT, thereby inhibiting the cytotoxic activity of NK cells and T cells (Gur et al., 2015). An example of the fourth mechanism, upregulation of immune checkpoint molecule expression, is the immune evasion of gastric cancer promoted by *H. pylori* CagA-mediated upregulation of PD-L1 levels in exosomes (Wang et al., 2023). The fifth mechanism, activation of immune suppressive cells, is exhibited by *Staphylococcus aureus*, HBV, HCV, and HPV, all of which promote the progression of prostate and liver cancer by inducing immune suppression mediated by Tregs (Adurthi et al., 2008; Ouaguia et al., 2019; Ma et al., 2020; Gao et al., 2022) (**Figure 2**).

## 6 Immunoregulation of the intratumoral microbiota in human cancers

There is significant heterogeneity in the intratumoral microbiota across different tumor tissues, with distinct microbiota shaping unique TIME. In the next section, we elucidate the research progress on the influence of intratumoral microbiota on the immune responses of various tumor types and summarize their clinical applications (**Table 1**).

**Table 1:** Regulation and application of the intratumoral microbiota-driven immune responses used for cancer assessment and therapy.

Classification	Tumor type	Immunomodulatory mechanism	Microbiota features	Effect	Ref.
Cancer Theraphy	BC	Activate T cells	*Blautia, Ruminococcus, Faecalibacterium, Dorea, Tyzzerella, Roseburia*	Enhance immunotherapy response	(Wang et al., 2022)
	Melanoma	Activate T cells	*Lactobacillus reuteri*	Enhance immunotherapy response	(Bender et al., 2023)
	CRC	Improve the antigen-presenting of DCs	*Bifidobacterium*	Enhance immunotherapy response	(Shi et al., 2020)
	Melanoma	Activate T cells	*Aclinetobacter, Actinomyces, Comamonas, Corynebacterium, Enterobacter, Roseomonas, Streptococcus*	The target of immunotherapy in different patients	(Kalaora et al., 2021)
	CRC	Immune gene mutation	*Dialister, Casaltella*	Evaluate survival in patients	(Byrd et al., 2023)
	CRC	Facilitate the immune surveillance of T cells	*Lachnospiraceae*	Inhibit cancer development	(Zhang et al., 2023)
	PDAC	Activate T cells , Upregulate PD-1 expression	*Proteobacteria , Bacteroidetes , Firmicutes*	Enhance immunotherapy response	(Pushalkar et al., 2018)
	GC	T cell activation, Upregulate PD-1 and CTLA-4 expression	Epstein-Barr virus	Enhance immunotherapy response	(Panda et al., 2018)
	CRC	Promote chronic inflammation	*F. nucleatum*	Evaluate prognosis in patients	(Yang et al., 2017)
Cancer Assessment	GC	Inactivate T cells	*Methylobacterium*	Evaluate prognosis in patients	(Peng et al., 2022)
	PC	Activate T cells	*Pseudoxanthomonas, Streptomyces, Saccharopolyspora, Bacillus clausii*	Evaluate survival in patients	(Riquelme et al., 2019)
	LC	Upregulate PD-1 expression	*Acinetobacter jungii*	Evaluate survival in patients	(Zhang et al., 2022)
	NPC	Inhibit T cells infiltration	*Corynebacterium, Staphylococcus*	Evaluate risk of malignant progression	(Qiao et al., 2022)
	Melanoma	Enhance T cells infiltration	*Lachnoclostridium, Flammeovirga*, *Gelidibacter, Acinetobacter*	Evaluate survival in patients	(Zhu et al., 2021)

BC, Breast cancer; GC, Gastric cancer; PC, Pancreatic cancer; LC, Lung cancer; CRC, Colorectal cancer; PDAC, Pancreatic ductal adenocarcinoma; NPC, Nasopharyngeal carcinoma.

### 6.1 Breast cancer

In comparison to healthy breast tissue, breast tumor tissues exhibit a reduced bacterial load, particularly with a notable deficiency in beneficial bacteria such as *Lactococcus* and *Streptococcus*. The deficiency weakens the antibacterial immune response, thereby facilitating the development of breast cancer (Xuan et al., 2014). A comprehensive case-control study involving 2,266 patients with primary, invasive breast cancer and 7,953 healthy women demonstrated that prolonged cumulative use of antibiotics is associated with an increased risk of breast cancer incidence and mortality. The correlation is likely due to bacterial dysbiosis, which diminishes bacteria-dependent immune cells (Velicer et al., 2004). Tzeng et al. discovered a deficiency of *Propionibacterium* in breast cancer. They reasoned that, because the abundance of this bacteria is positively correlated with the expression of genes related to T cells activation, the absence of *Propionibacterium* may promote tumor growth by inhibiting local T cells immunity (Tzeng et al., 2021). A balanced and diverse microbiota is likely to play a crucial role in maintaining immune surveillance and preventing cancer development. The absence of certain specific microorganisms could disrupt this balance, leading to impaired local immunity and potentially facilitating tumor growth. In the future, clinical researchers could explore treating breast cancer by orally administering beneficial bacteria to promote their migration to the mammary gland via the gut-breast axis. Alternatively, efforts could focus on directly transplanting beneficial bacteria into tumor tissues to enrich therapeutic approaches for breast cancer. The influence of bacterial metabolites in breast cancer tissues on immunity and the efficacy of immunotherapy has garnered increasing attention. In patients with triple-negative breast cancer (TNBC), the Clostridiales-related metabolite trimethylamine N-oxide (TMAO) was found to induce pyroptosis in tumor cells by activating the endoplasmic reticulum stress kinase PERK, thereby enhancing CD8+ T cell-mediated antitumor immunity (Wang et al., 2022).

### 6.2 Lung cancer

It is currently believed that the microbiota in lung cancer primarily influences tumor progression by altering the TIME and modulating local immune responses. Chronic inflammation induced by intratumoral bacteria can promote the growth and metastasis of lung cancer (Sommariva et al., 2020). Early epidemiological studies have indicated that bacterial infections are commonly present in lung cancer cases, negatively impacting lung cancer treatment and overall patient survival. Utilizing advanced high-throughput sequencing technologies, an increasing number of studies have demonstrated a correlation between local microbial dysbiosis and lung cancer (Qiao et al., 2015; Perez-Cobas et al., 2023). Jin et al. showed that local commensal bacteria in the lung stimulate bone marrow cells to produce Myd88-dependent IL-1β and IL-23, which induce the proliferation and activation of Vγ6+Vδ1+γδ T cells, leading to the production of IL-17 and other effector molecules, thereby promoting inflammation and tumor cell proliferation (Jin et al., 2019). Antibiotic aerosol inhalation therapy has been shown to reduce the number of bacteria in the lungs of mice, activate tumor-infiltrating T cells and NK cells, decrease the number of immunosuppressive Tregs, and enhance local antitumor immune responses (Le Noci et al., 2018).

### 6.3 Colorectal cancer

CRC tissues exhibit enrichment of *Fusobacterium* species. Research has shown that *F. nucleatum* can bind and activate the human inhibitory receptor CEACAM1 to inhibit the activities of T cells and NK cells, suggesting that CEACAM1 inhibitors could be used to treat *Fusobacterium*-colonized CRC (Gur et al., 2019). Many CRC researchers have focused on the interaction mechanisms between the gut microbiota and host metabolism. An integrated analysis of single-cell transcriptomics, microbiomics, metabolomics, and clinical cohort data of colorectal adenomas and CRCs confirmed that, during the progression from colorectal adenoma to CRC, there is a loss of gut symbiotic bacteria with urease activity, such as *Bifidobacterium*. This promotes the transition of macrophages to an immunosuppressive subtype, thereby promoting the development of CRC (Chen et al., 2023). Galeano Nino et al. discovered using spatial transcriptomics that, although CRC tissues contain a variety of bacteria, their distribution is uneven. Tumor regions colonized by bacteria exhibit high immunosuppressive activity, have fewer antitumor T cells compared to other regions, and show upregulated expression of immune checkpoint molecules, inhibiting T cells activity. This may help explain how the intratumoral microbiota of cancer patients influences the efficacy of immune checkpoint inhibitors (ICIs) (Galeano Nino et al., 2022). Mima et al. analyzed clinical data from 598 CRC samples and found that the amount of *F. nucleatum* in tumor tissues is negatively correlated with the density of CD3+ T cells, suggesting that *F. nucleatum* may promote the development of CRC by downregulating T cells-mediated adaptive immunity (Mima et al., 2015).

### 6.4 Pancreatic cancer

The microbiota in pancreatic cancer tissues exerts a carcinogenic effect by influencing the host immune system. Riquelme et al. discovered that the intratumoral microbiota of long-term survivors of pancreatic cancer was significantly enriched with *Pseudoxanthomonas*, *Streptomyces*, *Saccharopolyspora*, and *Bacillus clausii*. Furthermore, the two most abundant bacterial species identified in the tumors of long-term survivors reportedly possess immunoregulatory functions (Riquelme et al., 2019). *Porphyromonas gingivalis* promotes pancreatic cancer progression by creating an inflammatory microenvironment through the recruitment of neutrophils that release neutrophil elastase (Tan et al., 2022). Pushalkar et al. found that, compared to normal pancreatic tissue, both murine and human PDAC tissues possess a significantly more abundant microbiota, producing a tolerogenic immune program via selective activation of specific TLRs in monocytes (Pushalkar et al., 2018). Another noteworthy microbial group in pancreatic cancer is fungi, which have recently been reported to play a critical role in tumor formation. Aykut et al. demonstrated that *Malassezia* spp. are abundant in invasive PDAC tissues, promoting pancreatic cancer formation through activation of mannose binding lectin (Aykut et al., 2019).

## 7 Clinical application of the intratumoral microbiota in immunotherapy

The clinical efficacy of ICBs in solid tumors is impressive; however, there is significant variability of efficacy among different patients and cancer types (Helmink et al., 2019; Xie et al., 2022). The intratumoral microbiota has emerged as an important factor influencing ICB response, potentially through mechanisms such as infiltration and activation of intratumoral CD8+ T cells and upregulated expression of PD-L1. A study found that patients with metastatic gastric cancer benefited from treatment with the PD-L1 antibody avelumab, possibly attributable to higher levels of lymphocyte infiltration (Panda et al., 2018). Recent research demonstrated that gut-derived *Lactobacillus reuteri* migrates to the tumor site and produces I3A in an AhR-dependent manner, thereby inducing the cytotoxic activity of CD8+ T cells and enhancing the efficacy of anti-PD-L1 therapy (Bender et al., 2023). Anker et al. reported that a patient-derived prostate-specific microbe, CP1, possesses local immunostimulatory properties and can be used to reprogram a “cold” TIME, sensitizing it to anti-PD-1 immunotherapy and improving therapeutic outcomes (Anker et al., 2018). The characteristics of the intratumoral microbiota can also serve as prognostic biomarkers for predicting patient responses to ICB treatment. Vetizou et al. found that the antitumor effects of CTLA-4 blockade in melanoma patients depend on the type of *Bacteroides* species present (Vetizou et al., 2015).

Certain intratumoral microbiota promote the formation of an suppressive TIME, leading to the development of drug resistance. This microbial influence can be mitigated through antibiotic therapy. During CRC treatment, *F. nucleatum* predominantly invades the hypoxic interior of colorectal tumors, causing the tumor growth rate in mice to surge by 30-fold. Huang’s team developed a novel antibiotic, LipoAgTNZ, whose core component is a silver-tinidazole complex encapsulated in nanoliposomes for precise delivery to the tumor site. LipoAgTNZ enhances the antitumor immune response by increasing CD3+CD8+ T cells and CD44+CD62+ memory T cells, while reducing immunosuppressive tumor-associated M2 macrophages. Treatment with LipoAgTNZ rapidly eradicates colonizing microbiota, such as *F. nucleatum* and *E. coli* Nissle, leading to a long-term survival rate of 71% in CRC-bearing mice, which is significantly higher than that in the control group (Wang et al., 2023). Geng et al. prepared antibiotic-delivering nanocarriers that precisely target breast cancer tissues and effectively eliminate intratumoral *F. nucleatum* without disrupting the diversity and abundance of the systemic microbiota. This ultimately reprograms the TIME, improving the efficacy of PD-L1 blockers. This approach led to a tumor inhibition rate exceeding 90% and significantly extended the median survival of 4T1 tumor-bearing mice (Geng et al., 2024). Nevertheless, microbiota dysbiosis resulting from antibiotic therapy can be a long-term issue, persisting after treatment ends and not always easily reversed or corrected. Therefore, the pros and cons of antibiotic use must be carefully weighed, especially in long-term and immunotherapy-related treatments.

As a crucial component of the TIME, the intratumoral microbiota has potential for the development of novel diagnostic or prognostic markers. In 2020, two extensive studies examined the intratumoral microbiota across more than 30 cancer types. Riquelme et al. using targeted 16S rRNA amplicon sequencing of tumor DNA samples from pancreatic adenocarcinoma patients with different survival outcomes, discovered that long-term survivors (overall survival ≥ 5 years) had higher intratumoral microbial diversity than short-term survivors. They identified a signature feature of the microbiota, namely *Pseudoxanthomonas-Streptomyces-Saccharopolyspora-B. clausii*, that was highly predictive of long-term survival, indicating that the intratumoral microbiota might serve as a prognostic tool for determining patient survival (Riquelme et al., 2019). A study on the intratumoral microbiota of 802 nasopharyngeal carcinoma (NPC) patients showed that the tumor tissues were predominantly colonized by *Corynebacterium* and *Staphylococcus*. Patients with a higher bacterial load had lower disease-free survival rates and a negative correlation with T cells infiltration, suggesting that intratumoral bacterial load could be a powerful prognostic tool (Qiao et al., 2022). Ghaddar et al. identified tumor-associated bacterial subgroups related to cancer characteristics and immune activity that can be used to predict clinical prognosis and manage clinical outcomes in pancreatic cancer (Ghaddar et al., 2022).

Based on the selective colonization characteristics of microbiota in different tumor tissues, intratumoral microbiota can also serve as vectors to target tumors, delivering drugs (e.g. immunomodulators, ICIs, antibiotics) for precise tumor eradication. Tal Danino’s team constructed a genetically engineered strain of *E. coli* named “SLIC” that produces monoclonal antibodies targeting PD-L1 and CTLA-4, thereby activating T cells to attack cancer cells (Gurbatri et al., 2020). This team also designed a non-pathogenic strain of *E. coli* that specifically lyses within tumors and releases CD47 monoclonal antibodies, enhancing the activation of tumor-infiltrating T cells and improving the survival of tumor-bearing mice (Chowdhury et al., 2019). Canale et al. utilized synthetic biology to develop an engineered probiotic strain of *E. coli* Nissle 1917 that colonizes tumors and secretes L-arginine, thereby increasing the number of tumor-infiltrating T cells (Canale et al., 2021). Zhu et al. developed a probiotic food-grade *Lactococcus lactis*-based vaccination (FOLactis), which leads to significant tumor regression by increasing the number of conventional type 1 DCs in the TIME and restoring CTL responses. More importantly, it can synergize with PD-1 inhibitors to convert “cold tumors” into “hot tumors” (Zhu et al., 2022).

## 8 Future perspectives and challenges

Significant progress in elucidating the role of intratumoral microbiota in tumor immunity have uncovered therapeutic mechanisms and inspired the development of strategies for diagnosing and treating cancer by targeting these microbiota. These insights pave new avenues for personalized cancer therapy. Immune-regulating metabolites within the microbiota, such as microbial peptides, are abundantly present in the TIME, eliciting robust local and systemic immune responses. These microbial metabolites enhance tumor antigenicity and bolster tumor immune responses, suggesting their potential future application as tumor vaccines or adjuvants for tumor eradication. Although immunotherapy is a potent modality for combating tumors, it is imperative to assess the feasibility of immunotherapeutic regimens by monitoring each patient’s immune system characteristics before or during treatment. The TIME is crucial for tumor maintenance and therapeutic response, and the intratumoral microbiota, as a key component of TIME, significantly regulate the tumor immune milieu. Therefore, to systematically evaluate and optimize immunotherapy regimens, the impact of intratumoral microbiota on tumor immune responses should be incorporated into patient immune monitoring.

Molecular subtyping of tumors is fundamental for achieving precise cancer treatment. Over the past few decades, next-generation sequencing technologies have provided mutation data on the nucleic acids, proteins, and epigenetics of tumor tissues. These studies have significantly enhanced the understanding of tumor heterogeneity and expanded the methodologies for tumor classification. With continuous advancements in detection sensitivity and a deeper comprehension of tumors and their microenvironment, the dimensions of tumor classification have substantially broadened. There exists considerable compositional heterogeneity in the intratumoral microbiota across different tumor types and individual patients, which may emerge as a novel clinical pathological feature. In the future, intratumoral microbial signatures may serve as potential markers for tumor classification, thereby guiding diagnostic and therapeutic strategies and prognostic evaluation. Although recent achievements in correlating tumor microbiota with tumor immunity have not yet been widely implemented, it is anticipated that targeted interventions and predictive analyses of specific intratumoral microbiota will optimize immunotherapy, enhance treatment efficacy, and contribute to the development of more precise cancer therapies.

The influence of the intratumoral microbiota on the host immune system is profoundly intricate, with multifaceted interactions that need to be meticulously elucidated to enhance the efficacy of immunotherapy. Presently, this is an emerging field beset by numerous challenges. Firstly, the biological composition of the intratumoral microbiota is highly complex, displaying significant variability across different tumor types, individuals, and even within distinct regions of the same tumor. Host factors, including genetic background, lifestyle, medication usage, and immune status, exert substantial influence on the tumor microbiota, affecting both its composition and functional mechanisms, thereby compounding the complexity of research. This complexity poses a formidable challenge in comprehending how the intratumoral microbiota modulates the TIME and subsequent treatment responses. Secondly, although high-throughput sequencing technologies can provide extensive data regarding the characteristic of the intratumoral microbiota, there remain significant limitations in terms of sensitivity, specificity, and quantitative accuracy. The regulatory role of the intratumoral microbiota on the immune system holds immense potential for tumor diagnosis and prognostic evaluation and may be particularly instrumental in enhancing the efficacy of tumor immunotherapy. However, overcoming the aforementioned challenges and transforming research achievement to effective treatment strategies will require technological advancements and rigorous clinical validation.

## Author contributions

WL: Writing – original draft, Writing – review & editing. YL: Validation, Writing – original draft. PW: Writing – review & editing. XG: Writing – review & editing. YX: Writing – original draft. LJ: Supervision, Writing – original draft, Writing – review & editing. DZ: Supervision, Validation, Writing – original draft, Writing – review & editing.
